The article "Subclinical Diabetic Peripheral Vascular Disease and Epidemiology Using Logistic Regression Mathematical Model and Medical Image Registration Algorithm" was published in 2022. Journal: J Healthc Eng.

# Subclinical Diabetic Peripheral Vascular Disease and Epidemiology Using Logistic Regression Mathematical Model and Medical Image Registration Algorithm

**DOI:** 10.1155/2022/2116224

**Published:** 2022-01-17

**Authors:** Nailong Jia, Long Fan, Chuizhi Wang, Qimao Fu, Yan Chen, Changkun Lin, Yupeng Zhang

**Affiliations:** Department of Radiology, The Second Affiliated Hospital of Hainan Medical College, Haikou 570311, Hainan, China

## Abstract

The study aims to explore the effect of subclinical diabetic peripheral vascular disease and an epidemiological investigation of colour Doppler ultrasound images based on a logistic regression mathematical model and a medical image registration algorithm. Subclinical diabetes patients were selected as subjects, and after ultrasound colour Doppler ultrasonography of peripheral blood vessels, ultrasound images were taken. The experimental results show that the area under the curve (AUC) predicted by the model was 0.748, the sensitivity was 94.12%, and the specificity was 67.93%. All Δ were smaller than a single pixel. The detection rate of colour Doppler ultrasonography was 82.6%, which was significantly better than that of clinical examination (*P* < 0.01). The age, course of disease, SBP, low-density lipoprotein cholesterol (LDL-C), total cholesterol (TC), and triglyceride (TG) of the peripheral vascular disease group were significantly different from those of the no peripheral vascular disease group (*P* < 0.05). The incidence of peripheral vascular diseases and nonperipheral vascular diseases in male patients was remarkably higher than that in female patients (*P* < 0.05). Moreover, with the increase of age, the incidence of peripheral vascular disease and nonperipheral vascular disease in diabetic patients showed a trend of gradual increase (*P* < 0.05). In summary, the mathematical model and registration method have high accuracy for medical image registration of patients with the diabetes epidemic. In addition, the age, course of disease, SBP, LDL-C, TG, and TC of diabetic patients were significantly different from those of normal people, which can provide a reference for the development of later diabetes epidemiology.

## 1. Introduction

When doctors diagnose and treat patients' diseases, they often need to image patients with X-ray, CT, MRI, PET, SPECT, and other imaging modes to provide complementary information on patient anatomy and functional metabolism. Multimode medical image registration is to transform the spatial position of pixels in an image so that it is aligned with the pixels of other pattern images in spatial position, thereby merging image data of various imaging modes and utilizing respective image information [1]. The characteristic is to express information from many aspects of the human body on an image. The voxel similarity-based registration method is a method of high precision and robustness because it directly uses the statistical property of image pixel grayscale information, i.e., mutual information, as the basis for registration, without extracting the anatomical features of the image. Compared with the traditional method, this method has the advantages of high registration accuracy (reaching subturbulence level), good reliability, and no need for image presegmentation and feature extraction. The image after registration and fusion is more conducive to further clinical comprehensive diagnosis [2]. It has received widespread attention and has found wide application in the field of medical image registration.

The article "Subclinical Diabetic Peripheral Vascular Disease and Epidemiology Using Logistic Regression Mathematical Model and Medical Image Registration Algorithm" was published in 2022. Journal: J Healthc Eng.

The most used optimization algorithms in mutual information-based medical image registration are the simplex method and the Powell method, in addition to the simulated annealing algorithm and the genetic algorithm [3]. These optimization algorithms have their own advantages, but they all have shortcomings. The Powell method and the simplex method do not need to calculate the derivative, but the Powell method can easily fall into the local optimum in the registration process, while the simplex method converges too slowly; the simulated annealing algorithm can jump out of the local optimal trap. The time is long and sometimes enters the wrong search direction, so the optimal solution cannot be obtained, and the genetic algorithm is prone to the problem of “premature convergence” [4].

As China continues to age, the incidence of diabetes epidemiology is on the rise, and peripheral vascular disease is the main cause of disability in subclinical diabetes. Clinically, when there are obvious symptoms, it indicates that peripheral vascular lesions have occurred for macrovascular disease. 190 cases of subclinical diabetes epidemic patients in our hospital were examined by colour Doppler ultrasound. A binary logistic regression mathematical model was established to analyze the fitting effect, and a mutual information medical image registration algorithm was used for image analysis. The objective is to know the pathological changes and epidemiological characteristics of peripheral blood vessels more accurately in patients with diabetes mellitus and to explore the risk factors of pathological changes for early diagnosis and prevention.

## 2. Data and Methods

### 2.1. General Information

In this study, 190 cases of subclinical diabetes epidemic patients were selected from October 2017 to October 2020. The selected patients met the WHO criteria for diabetes diagnosis, including renal dysfunction, myocardial infarction, cerebral haemorrhage, and cerebral infarction. There were 130 males and 60 females, aged 38–79 years old, with an average of (58.9 ± 6.9) years. The course of disease was 1–28 years, with an average of (7.1 ± 3.4) years. Another 33 healthy subjects were selected as the group without peripheral vascular disease. The patients included had signed informed consent, and the study had been approved by the ethics committee of the hospital.

The article "Subclinical Diabetic Peripheral Vascular Disease and Epidemiology Using Logistic Regression Mathematical Model and Medical Image Registration Algorithm" was published in 2022. Journal: J Healthc Eng.

### 2.2. Research Methods

#### 2.2.1. Laboratory Inspection

All patients were fasting venous blood on the 2nd day after admission and were checked for fasting blood glucose (FBG), glycosylated hemoglobin (HbAlc), low-density lipoprotein cholesterol (LDL-C), high-density lipoprotein cholesterol (HDL-C), total cholesterol (TC), and triglyceride (TG).

#### 2.2.2. Colour Doppler Ultrasonography

Using the colour Doppler diagnostic instrument, the probe frequency was 7.5∼10.0 MHz, the wall filter was 50∼100 Hz, and the angle between the sound beam and the blood flow was <60°. The patient was placed in the supine or prone position, and the feet were straightened. The bilateral peripheral arterial vessels (femoral common femoral artery, superficial femoral artery, deep femoral artery, radial artery, dorsal artery, and anterior tibialis anterior artery) were examined to detect the diameter of the vessel. Intravascular wall plaque, observing vascular stenosis and colour flow filling, measuring intravascular-medial thickness (IMT). The diagnostic criteria for peripheral vascular disease are as follows: stenosis; plaque (single, multiple, and diffuse); intima is not thick, but echo is enhanced; femoral artery IMT ≥1 mm.

## 3. The Registration Method Based on Mutual Information and the Hybrid Optimization Algorithm

### 3.1. Image Registration Principle Based on Mutual Information

Mutual information is a basic concept in information theory. It is used to describe the statistical correlation between two random variables. It can be described by entropy as follows:

(1) $$\begin{array}{c} I\left(A,B\right)=H\left(A\right)+H\left(B\right)-H\left(A,B\right). \end{array}$$

### 3.2. Registration Transformation Model

For the two images to be registered, a unified stereo coordinate system is first established. The coordinate origin is defined in the gravy centre of gravity of the image, and the two images are coarsely registered. Selecting one image as the reference image *R* and the other image as the floating image *F*, the rigid body transformation from the spatial coordinate PF of the floating image to the spatial coordinate PR of the reference image can be described by the following equation:

(2) $$\begin{array}{c} V_{R}\circ \left(P_{R}-C_{R}\right)=R_{x}\left(\Phi_{x}\right)\circ R_{y}\left(\Phi_{y}\right)\circ R_{z}\left(\Phi_{z}\right)\circ V_{F}\circ \left(P_{F}-C_{F}\right)+t\left(t_{x},t_{y},t_{z}\right). \end{array}$$

The article "Subclinical Diabetic Peripheral Vascular Disease and Epidemiology Using Logistic Regression Mathematical Model and Medical Image Registration Algorithm" was published in 2022. Journal: J Healthc Eng.

### 3.3. Hybrid Optimization Algorithm

The genetic algorithm (GA) is an efficient parallel global search algorithm that simulates the principle of natural selection and genetic mechanism. The GA algorithm flow is shown in Figure 1. Unlike many traditional search algorithms, the search results are closely related to the initial point selection and are easy to fall into the local maximum excellent solution [5].

The SA starts from a higher initial temperature *T*, and with the continuous decrease of the temperature parameter, the probability of the jump feature is combined with the global optimal solution of the objective function in the solution space; that is, the local optimal solution jumps probabilistically and finally tends to be globally optimal [6]. The SA algorithm flow is shown in Figure 2.

The scope of the search will be narrowed rapidly, but the rapidly converged group does not necessarily achieve the global optimal, which leads to the problem of “premature convergence” [7]. For this “premature convergence,” a hybrid optimization algorithm combining the genetic algorithm and the simulated annealing algorithm is an effective solution to introduce Metropolis acceptance criteria in GA.

### 3.4. Hybrid Optimization Algorithm Parameter Determination

(1) In the implementation of the hybrid optimization algorithm, the gene population with the number of chromosomes *n* = 50 is selected, the gene string length is 57, the coding order is (*t*_*x*_, *t*_*y*_, *t*_*z*_, Φ_*x*_, Φ_*y*_, Φ_*z*_), the single-point crossover is adopted, the crossover probability is 0.6, and the mutation probability is 0.02.
Each parameter in the stiffness transformation parameter (*t*_*x*_, *t*_*y*_, *t*_*z*_, Φ_*x*_, Φ_*y*_, Φ_*z*_) is encoded. Since, the coordinate centre of the image is defined in the gravy centre of gravity of the image, which is equivalent to coarse registration of the two images, the amount of translation in the direction of the coordinate axis is generally not large, between −15 and 15 mm, each translation parameter uses 9-bit binary code, the rotation angle is between −10° and 10°, each translation parameter uses 10-bit binary code, so the resolution of the translation amount is about 0.06 mm/bit, and the resolution of the angle is about 0.02°/bit.
(2) In order for the algorithm to reach a quasiequilibrium state at the beginning, the initial acceptance rate should be made.
  (3) $$\begin{array}{c} \chi_{0}=\frac{M}{N}\approx 1. \end{array}$$

In this study, it uses the method proposed in [8] to determine *T*_0_ by calculating the average increment of the objective function of several random transformations:

(4) $$\begin{array}{c} T_{0}=\frac{\overset{——}{\Delta f^{+}}}{\ln\left(\chi_{0}^{-1}\right)}. \end{array}$$

The overall structure of mutual information hybrid algorithms is shown in Figure 3.

The article "Subclinical Diabetic Peripheral Vascular Disease and Epidemiology Using Logistic Regression Mathematical Model and Medical Image Registration Algorithm" was published in 2022. Journal: J Healthc Eng.

### 3.5. Applying a Hybrid Optimization Algorithm to Solve Spatial Transformation Parameters

The main steps of applying mutual information and hybrid optimization algorithms for image registration are as follows:

(1) Initialize the parameters of the algorithm, *T* ⟶ *T*0, randomly generate a group of initial individuals to form the initial population, and calculate the corresponding objective function value *f* of everyone in the population, called the fitness value. The individual fitness value of everyone in this study is individual. Mutual information minus the minimum mutual information in this generation of individuals;
(2) Determine whether the algorithm stops the criterion. If it is met, the algorithm ends and returns the optimal solution; otherwise, the following steps are performed;
(3) Using the roulette method to select n/2 pairs of individuals with large adaptation values from the population, as the parent, perform the following operations for each pair of parents:
    (a) Calculate the fitness value *f*_*C*1_, *f*_*C*2_ of C1, C2 by the parent P1, P2 by crossing and mutating to generate the children C1, C2
    (b) If *f*_*Ci*_(*f*_*Pi*_, (*i*=1,2)), replace Pi with Ci; otherwise, accept Ci with probability exp[−(*f*_*Ci*_ − *f*_*Pi*_)/*T*]
(4) *T*=*T*∘*α*, return 2.

## 4. CT-MR Registration

The Vanderbilt University “Review Image Registration Algorithm Evaluation” project has a set of subclinical diabetes patient data practice groups for researchers to conduct initial evaluation of the algorithm. The data set for CT-MR and PET-MR registration is also given. As a result, we applied this set of data and its standard results to evaluate the accuracy of the algorithm results.

The practice group includes a set of CT data and 6 sets of MR data for a subclinical diabetic patient. The 6 sets of MR data are PD, T1, T2, and PD-rectified, T1-rectified, and T2-rectified images, respectively. CT image resolution is 512 × 512 × 29 and voxel size is 0.653595 mm × 0.653595 mm × 4 mm. MR image resolution is 256 × 256 × 26, and voxel size is (1.25∼1.28 mm) × (1.25∼1.28 mm) × (4∼4.12 mm).

We use the registration method proposed in this study to register CT and MRI images, using MRI images as registration reference images, CT images as registration floating images, and the PV interpolation method for registration experiments. In the experiment, the image data is subsampled to speed up the calculation, and the sampling range on the XY plane is limited to the centre of gravity of the human brain, which reduces the influence of image background pixels on mutual information calculation. We evaluate the accuracy of the registration results by the following methods: 8 vertices qi, MI of the registered floating image, and 8 vertices *q*_*i*,ref_ of the standard result:

(5) $$\begin{array}{c} \Delta =\frac{1}{8}\sum_{i=1}^{8}\left|q_{i,\mathrm{ref}}-q_{i,\mathrm{MI}}\right|, \end{array}$$

(6) $$\begin{array}{c} \Delta k=\frac{1}{8}\sum_{i=1}^{8}\left|\sum_{i=1}^{8}\left|q_{i,\mathrm{ref},k}-q_{i,\mathrm{MI},k}\right|\right|k=x,y,z, \end{array}$$

where Δ represents the average geometric distance of the eight corresponding vertices, representing the average absolute error along the coordinate axis, and the registration results are compared with the gold standard according to equations (5) and (6). The results are shown in Table 1.

The article "Subclinical Diabetic Peripheral Vascular Disease and Epidemiology Using Logistic Regression Mathematical Model and Medical Image Registration Algorithm" was published in 2022. Journal: J Healthc Eng.

The registration results of the first 4 behaviours in the table and the registration result of the 5th behaviour document are shown. The pixel diagonal distance in the *M* R image is taken as a pixel size, namely:

(7) $$\begin{array}{c} \sqrt{1.25^{2}+1.25^{2}+4.0^{2}}\approx 4.373\mathrm{mm}. \end{array}$$

It can be concluded from Table 1 that all Δ are smaller than a single pixel size, and our registration result meets the subpixel precision requirement. The characteristics of the data are used to set the transformation parameter search order in the Powell optimization process. However, the algorithm does not make any assumptions about the image data of the test. It is not necessary to modify the optimization process for the characteristics of the image. Overall, our algorithm's registration result is better, and the versatility is stronger.

Figure 4 shows the CT image and MR image of the patient in the practice group and the registration results. Comparing Figures 1(a) and 1(b), the original spatial positions of the two images differ greatly. From (d), after the transformation, the two images achieved a good registration result.

## 5. Statistical Analysis

The results were expressed as mean ± standard deviation (*x* ± *s*), and SPSS25.0 statistical software was used for statistical analysis. The incidence rate of peripheral vascular disease and nonperipheral vascular disease was observed by the rank sum test. The results of two groups were compared by the *t* test and the *x*^2^ test. *P* < 0.05 showed that there was statistical difference, and *P* < 0.01 indicated significant statistical difference. The binary logistic regression model was established according to the single factor. The Hosmer–Lemeshow goodness-of-fit test was used to evaluate the fitting degree of the model. The accuracy of the prediction model was evaluated by AUC (area under the curve).

The article "Subclinical Diabetic Peripheral Vascular Disease and Epidemiology Using Logistic Regression Mathematical Model and Medical Image Registration Algorithm" was published in 2022. Journal: J Healthc Eng.

## 6. Results

### 6.1. Colour Doppler Ultrasonography for Peripheral Vascular Disease

Among 190 patients, 157 cases of peripheral vasculopathy were detected by colour Doppler ultrasound, including 132 cases of plaque, accounting for 84.1%; 64 cases of intimal thickening, accounting for 40.8%; and 38 cases of arteriosclerosis, accounting for 24.2%. There were 32 cases of vascular stenosis, accounting for 20.4%, and 16 cases of vascular occlusion, accounting for 10.2%. 105 cases of the posterior tibial artery were involved, accounting for 66.9%; 90 cases of the dorsal artery, accounting for 57.3%; 65 cases of the femoral artery, accounting for 41.4%; 54 cases of the anterior tibial artery, accounting for 34.4%; and 40 cases of radial artery 6, accounting for 25.5% (Figures 5 and 6).

### 6.2. Comparison of Clinical Examination and Colour Doppler Ultrasonography

Among the 190 patients, 56 patients had symptoms (peripheral limb pain, numbness, peripheral cold sensation, foot ulcer, and dorsal artery pulsation disappeared). The detection rate was 29.5%; colour Doppler ultrasonography showed there were 157 cases of peripheral vascular disease, and the detection rate was 82.6%; the detection rate of the latter was significantly better than the former, and the difference was statistically significant (*P* < 0.01).

### 6.3. Analysis of Peripheral Vascular Disease Factors

The age, duration of disease, SBP, LDL-C, TG, and TC in the group with peripheral vascular disease were significantly different from those without peripheral vascular disease (*P* < 0.05 or < 0.01). There were no significant differences in gender, BMI, DBP, FBG, HbAlc, and HDL-C between the patients with peripheral vascular disease and those without peripheral vascular disease (*P* > 0.05) (Table 2).

### 6.4. Epidemiological Analysis of Peripheral Vascular Diseases of Different Ages and Genders

The incidence of peripheral vascular disease and nonperipheral vascular disease was compared in diabetic patients of different ages and genders (Table 3). It was found that the incidence rate of peripheral vascular disease and nonperipheral vascular disease in male patients were higher than that in females, and the difference was statistically significant (*P* < 0.05). With the increase of age, the incidence rate of peripheral vascular disease and nonperipheral vascular disease in diabetes showed a gradual increase trend (*P* < 0.05).

The article "Subclinical Diabetic Peripheral Vascular Disease and Epidemiology Using Logistic Regression Mathematical Model and Medical Image Registration Algorithm" was published in 2022. Journal: J Healthc Eng.

### 6.5. Analysis of Prediction and Fitting Effects of the Mathematical Model

The meaningful independent variables were selected, and the ROC curve of the mathematical model constructed is shown in Figure 7. Through repeated calculation, the AUC value predicted by the model was 0.748, the sensitivity was 94.12%, and the specificity was 67.93%, which indicated that the logistic regression model had a good fitting effect.

## 7. Discussion

Subclinical diabetic peripheral vascular disease is a common complication of diabetes, and severe cases can cause gangrene in patients. According to statistics, the amputation rate of diabetic peripheral vascular disease is 5 to 10 times that of normal people, and the incidence of peripheral vascular disease with a diabetes duration of more than 5 years is more than 90%, while that of nondiabetics is 10%. The early clinical manifestations of peripheral vascular disease lack specificity. Once there is resting pain, intermittent claudication, ischemic gangrene, etc., trauma treatment or amputation is needed, which brings psychological and physiological relief to the patient. The pain also increases the pressure on the patient's life [10]. Diabetes epidemiology was investigated, and the results showed that the incidence rates of peripheral vascular disease and nonperipheral vascular disease in male diabetic patients were higher than those in females (*P* < 0.05), and the incidence rates of prediabetes and diabetes increased gradually with age, which was consistent with the results of [11]. Therefore, the early diagnosis and prevention of subclinical diabetes and peripheral vascular disease is particularly important.

Colour Doppler ultrasonography is characterized by simple operations and no trauma. It can detect arterial lesions early and make effective judgments on the severity of lesions and the location of lesions [12]. Research shows that colour Doppler ultrasound is the preferred method for peripheral vascular lesion examination in subclinical diabetes patients and has important clinical guiding significance for early diagnosis, prevention, and treatment. In this group of 190 patients with subclinical diabetes, the detection rate of peripheral vascular lesions was 29.5%, and colour Doppler ultrasonography was 82.6%. The detection rate of the latter was significantly better than the former. The difference was statistically significant (*P* < 0.01). Studies have shown that colour Doppler ultrasound examinations can be used as a routine examination of T2DM, which is conducive to the early detection of peripheral vascular lesions. Among the 157 patients with peripheral vascular disease, plaque accounted for 84.1%, followed by intima thickening in 64 cases. The cumulative posterior tibial artery was 66.9%, followed by the dorsal artery. Studies have shown that peripheral vascular lesions are mainly plaques, followed by intimal thickening, and cumulative after the posterior tibial artery. After the logistic regression mathematical model was constructed, the prediction fitting effect was good, which was consistent with the research of [13].

The article "Subclinical Diabetic Peripheral Vascular Disease and Epidemiology Using Logistic Regression Mathematical Model and Medical Image Registration Algorithm" was published in 2022. Journal: J Healthc Eng.

## 8. Conclusion

In this study, the hybrid optimization algorithm was used to register the multi-mode medical images. The genetic algorithm is a popular global optimization strategy with a wide application space. In addition, the algorithm also has good advancements, which can easily overcome the problem that the genetic algorithm is prone to early convergence, and it is not easy to fall into a local optimal state. The accuracy of the algorithm can reach subpixel levels, and the algorithm can be automatically implemented. This method is suitable for clinical application because it does not require manual intervention or more preprocessing of images. However, the theoretical derivation and model establishment need to be further discussed, and the registration accuracy also needs to be improved.

## Figures and Tables

**Figure 1:** Genetic algorithm flow.

**Figure 2:** Simulated annealing algorithm (SA) process.

**Figure 3:** Mutual information hybrid algorithms.

**Figure 4:** CT-MR image registration result.

**Figure 5:** Colour Doppler image of the anterior tibial artery.

**Figure 6:** Brachial artery colour Doppler images.

**Figure 7:** The ROC curve of the logistic regression mathematical model constructed.

**Table 1:** CT-MR registration results.

	CT-PD	CT-T1	CT-T2	CT-PDr	CT-T1r	CT-T2r
Δ*x*	0.723	1.212	2.083	1.561	0.407	1.169
Δ*y*	0.772	1.261	2.061	1.442	0.781	1.203
Δ*z*	1.712	1.190	2.330	2.600	1.129	1.251
Δ	2.210	2.262	3.891	3.818	1.535	2.350
Δ [9]	2.561	1.698	2.899	3.144	1.873	3.712

**Table 2:** Analysis of related factors in the groups with peripheral vascular disease and without peripheral vascular disease.

Index	Peripheral vascular disease group (*n* = 157)	Without peripheral vascular disease group (*n* = 33)	*χ* ^2^/*t*	*P*
Gender (male or female)	108/49	20/13	0.363	0.125
Age (years)	66.2 ± 6.6	51.8 ± 5.4	7.791	0.000
Disease course (years)	9.1 ± 2.5	5.5 ± 1.6	6.772	0.000
BMI (kg/m^2^)	24.1 ± 2.7	23.8 ± 2.2	0.547	0.120
SBP (mmHg)	160.4 ± 16.1	129.0 ± 14.9	7.039	0.000
DBP (mmHg)	78.2 ± 7.8	74.1 ± 6.2	0.993	0.088
FBG (mmol/L)	9.7 ± 2.5	9.6 ± 3.3	0.105	0.323
HbAlc (%)	8.2 ± 0.9	8.6 ± 1.0	1.326	0.072
HDL-C (mmol/L)	1.3 ± 0.5	1.4 ± 0.8	0.573	0.116
LDL-C (mmol/L)	2.9 ± 0.9	2.1 ± 1.0	2.674	0.063
TG (mmol/L)	2.6 ± 1.2	2.0 ± 1.8	2.558	0.069
TC (mmol/L)	5.6 ± 1.3	4.9 ± 0.7	2.373	0.072

The article "Subclinical Diabetic Peripheral Vascular Disease and Epidemiology Using Logistic Regression Mathematical Model and Medical Image Registration Algorithm" was published in 2022. Journal: J Healthc Eng.

**Table 3:** Comparison of the incidence of peripheral vascular disease and nonperipheral vascular disease in diabetic patients of different ages and genders (case (%)).

Age	Peripheral vascular disease (*n* = 157)			Nonperipheral vascular disease (*n* = 33)		
	Male	Female	Total	Male	Female	Total
30–40	8 (5.10)	7 (4.46)	15 (9.55)	3 (9.09)	1 (3.03)	4 (12.12)
40–50	12 (7.64)	10 (6.37)	22 (14.01)	3 (9.09)	2 (6.06)	5 (15.15)
50–60	18 (11.46)	13 (8.28)	31 (19.75)	4 (12.12)	2 (6.06)	6 (18.18)
60–70	24 (15.29)	16 (10.19)	40 (25.48)	5 (15.15)	3 (9.09)	8 (24.24)
70–80	29 (18.47)	20 (12.74)	49 (31.21)	7 (21.21)	3 (9.09)	10 (30.30)
*P*	0.001	0.002	0.001	0.01	0.03	0.001

## Data Availability

The data used to support the findings of this study are available from the corresponding author upon reasonable request.
